The article "Clinical Relevance of Anticoagulation and Dual Antiplatelet Therapy to the Outcomes of Patients With Atrial Fibrillation and Recent Percutaneous Coronary Intervention With Stent" was retracted in 2025. Reasons: duplicate publication; overlap with earlier publications.

# Clinical Relevance of Anticoagulation and Dual Antiplatelet Therapy to the Outcomes of Patients With Atrial Fibrillation and Recent Percutaneous Coronary Intervention With Stent

**DOI:** 10.14740/jocmr2443w

**Published:** 2015-12-28

**Authors:** Renato De Vecchis, Claudio Cantatrione, Damiana Mazzei

**Affiliations:** a Cardiology Unit, Presidio Sanitario Intermedio “Elena d’Aosta”, ASL Napoli 1 Centro, Napoli, Italy

**Keywords:** Atrial fibrillation, Percutaneous coronary intervention, Antithrombotic therapy, Major adverse cardiovascular events, Bleeding

## Abstract

**Background:**

Chronic atrial fibrillation (AF), coexisting with a history of recent coronary angioplasty with stent (PCI-S), represents an encoded indication for oral anticoagulation (OAC) with warfarin plus dual antiplatelet therapy (DAPT).

**Methods:**

Using a retrospective cohort study, we determined the respective impacts on cardiovascular outcomes of three different pharmacologic regimens, i.e., triple therapy (TT) with warfarin + clopidogrel and aspirin, dual therapy (DT) with warfarin + clopidogrel or aspirin, and DAPT with clopidogrel + aspirin. Outcomes of interest were all-cause mortality, ischemic cardiac events, ischemic cerebral events, and bleeding events. The inclusion criterion was the coexistence of an indication for OAC (e.g., chronic AF) with an indication for DAPT due to recent PCI-S.

**Results:**

Among the 98 patients enrolled, 48 (49%), 31 (31.6%), and 19 (19.4%) patients were prescribed TT, DT, and DAPT, respectively. Throughout a mean follow-up of 378 ± 15.7 days, there were no significant differences between the three regimens for all abovementioned outcomes. In particular, the total frequency of major bleeding was similar in the three groups: five cases (10.4%) in TT, one case (3.22%) in DT and no case in DAPT groups (Chi-square test, P = 0.1987).

**Conclusions:**

TT, DT and DAPT displayed similar efficacy and safety. Although the superiority of OAC vs. DAPT for stroke prevention in AF patients has been demonstrated by previous randomized trials, a smaller frequency of high thromboembolic risks’ features in DAPT group of the present study may have prevented the observation of a higher incidence of ischemic stroke in this group.

## Introduction

A condition commonly found in clinical practice is the coexistence of chronic or persistent atrial fibrillation (AF), which requires oral anticoagulation (OAC) [1] with angina pectoris or acute coronary syndrome (ACS), which requires percutaneous coronary intervention with stenting (PCI-S) [2], consistently followed by prolonged administration of dual antiplatelet therapy (DAPT) with acetylsalicylic acid (ASA) combined with another suitable platelet antiaggregant (e.g., a thienopyridine such as clopidogrel or prasugrel) [3]. The DAPT is less effective than the OAC in the conditions where the latter is indicated (e.g., chronic AF) [1]. By contrast, the OAC, even when associated with ASA, is less effective than DAPT to prevent intra-stent thrombosis or relapses of myocardial ischemia after PCI-S [2]. Thus, the combination of OAC and DAPT, a so-called “triple therapy” (TT), would seem to be the most rational solution for patients undergoing PCI-S for ACS or stable effort angina in whom an indication coexists for long-term OAC [4-8]. However, this TT with OAC, ASA, and clopidogrel is notoriously regarded to raise the opportunity for bleeding complications [8, 9].Thus, considering the very feared increase in bleeding inherent in the TT, experimental attempts have been made to reduce the risk of bleeding without diminishing the prophylactic effectiveness against AF-related cardioembolic events by adopting a simplified regimen, i.e., warfarin in combination with a sole antiplatelet agent (clopidogrel or ASA) [8, 10].

The article "Clinical Relevance of Anticoagulation and Dual Antiplatelet Therapy to the Outcomes of Patients With Atrial Fibrillation and Recent Percutaneous Coronary Intervention With Stent" was retracted in 2025. Reasons: duplicate publication; overlap with earlier publications.

The aim of this study was to make a comparative evaluation of the efficacy and safety endpoints of three different therapeutic strategies adopted within a population of patients, each of whom has a potential indication for both OAC and DAPT.

## Methods

Monocentric case records of outpatients with AF and history of previous PCI with implantation of one or more bare metal stent (BMS) or drug-eluting stent (DES) (either sirolimus or everolimus) were retrospectively examined. The timeframe taken into account spans from January 2008 to December 2013. Data concerning the patients included in our retrospective evaluation were taken from their electronic outpatient folders. Inclusion criterion was the documented indication for prophylaxis of thromboembolic events with warfarin (due to chronic or persistent AF, mechanical valve prosthesis, and deep vein thrombosis) accompanied by the simultaneous indication in the same patient for prevention of a possible post-procedural intra-stent thrombosis by means of DAPT (the latter being administered due to recent PCI-S procedure for angina or ACS). Furthermore, for admission into the study, regular administration for an adequate period (not less than 1 month) should have been documented, for one of the following drug regimens: 1) TT with warfarin plus the combination therapy with ASA and clopidogrel; 2) dual therapy (DT) with warfarin plus either ASA or clopidogrel (i.e., one only of the two above mentioned antiplatelet agents; or 3) DAPT with ASA and clopidogrel. Furthermore, in the case where AF had been the indication for OAC, patients in whom AF had begun before the coronary stent implantation were considered separately from patients in whom AF had occurred after the stent implantation. Because of the retrospective nature of our study, the investigators did not interfere in the selection of patients assigned to the three treatment regimens. The pharmacologic associations and their doses were determined for each patient, according to the full discretion of the treating physicians and based on criteria that included the patient’s general condition, comorbidities, and especially the profiles of both thrombotic and bleeding risk according to the CHA_2_DS_2_-VASc [11] and HAS-BLED [11] scores, respectively (explanatory synopses for both the scores shown in Tables 1 and 2). The data were meticulously collated and elaborated to build the summarizing tables.

The article "Clinical Relevance of Anticoagulation and Dual Antiplatelet Therapy to the Outcomes of Patients With Atrial Fibrillation and Recent Percutaneous Coronary Intervention With Stent" was retracted in 2025. Reasons: duplicate publication; overlap with earlier publications.

**Table 1:** CHA_2_DS_2_-VASc Score for Estimating the Risk of Stroke in Patients With Atrial Fibrillation

	Condition	Points
C	Congestive heart failure (or left ventricular systolic dysfunction)	1
H	Hypertension: blood pressure consistently above 140/90 mm Hg (or treated hypertension on medication)	1
A_2_	Age ≥ 75 years	2
D	Diabetes mellitus	1
S_2_	Prior stroke or TIA or thromboembolism	2
V	Vascular disease (e.g. peripheral artery disease, myocardial infarction, aortic plaque)	1
A	Age 65 - 74 years	1
Sc	Sex category (i.e. female sex)	1

The CHA_2_DS_2_-VASc score is a refinement of CHADS_2_ score and extends the latter by including additional common stroke risk factors, such as vascular disease, age 65 - 74 years and sex category (i.e. female sex). The maximum CHA_2_DS_2_-VASc score is 9 (for age, either the patient is ≥ 75 years and gets two points, is between 65 and 74 and gets one point, or is under 65 and does not get points). Note that female gender only scores one point if the patient has at least one other risk factor, and does not score any points in isolation. TIA: transient ischemic attack.

**Table 2:** HAS-BLED Score for Assessing the Bleeding Risk During Oral Anticoagulation Among Patients With AF

	Clinical feature	Points
H	Hypertension (systolic blood pressure > 160 mm Hg)	1
A	Abnormal renal function (defined as the presence of chronic dialysis or renal transplantation or serum creatinine ≥ 200 µmol/L (> about 2.3 mg/dL))	1
	Abnormal liver function (defined as chronic hepatic disease (e.g. cirrhosis) or biochemical evidence of significant hepatic derangement (e.g. bilirubin > × 2upper limit of normal, in association with AST/ALT/ALP > × 3 upper limit normal)	1
S	Stroke (previous history of stroke)	1
B	Bleeding (major bleeding history (anemia or predisposition to bleeding))	1
L	Labile INRs (refers to unstable/high INRs or poor time in therapeutic range (e.g. < 60%))	1
E	Elderly (age ≥ 65 years)	1
D	Drug therapy (concomitant therapy such as antiplatelet agents, NSAIDs, steroids)	1
	Alcohol intake (consuming 8 or more alcoholic drinks per week)	1
		Maximum score: 9 points

Risk of major bleeding: score 0 = 1%/year, score 5 = 12.5%/year. HAS-BLED score interpretation A score of 3 or more indicates an increased risk of bleeding that would be sufficient to justify the prudence or more frequent assessment. Physicians should also remember that the risk of bleeding may be changed and the HAS-BLED score can help you understand what correct: for example, discontinuation of therapy with aspirin and a better blood pressure control may be two ways to reduce the risk of bleeding. AST: aspartate aminotransferase; ALT: alanine aminotransferase; ALP: alkaline phosphatase; INR: international normalized ratio; NSAIDs: non-steroidal anti-inflammatory drugs.

The article "Clinical Relevance of Anticoagulation and Dual Antiplatelet Therapy to the Outcomes of Patients With Atrial Fibrillation and Recent Percutaneous Coronary Intervention With Stent" was retracted in 2025. Reasons: duplicate publication; overlap with earlier publications.

### Statistical analysis

All statistical tests were made with a commercially available statistical analysis program (SPSS 15.0 for Windows, SPSS Inc., Chicago, IL, USA). The distribution of the data was assessed using the D’Agostino-Pearson test. Continuous variables displaying normal distribution were expressed as mean ± SD, while values with asymmetric distribution were expressed as medians with interquartile ranges. Categorical variables were presented as percentages (%). The comparisons were made by means of the one-way analysis of variance (ANOVA) (continuous variables) or by applying the Chi-square test (categorical variables). The impact of the three antithrombotic therapies on several outcomes, such as major adverse cardiovascular events (MACEs), total bleeding, major bleeding events, and total events (MACEs plus bleeding) was evaluated with the Kaplan-Meier method, and differences between treatment groups were estimated with the log-rank test. Ethical approval was not requested, since it is usually not prescribed for retrospective cohort studies in Italy because patients cannot be identified.

## Results

In this study, 98 patients were retrospectively recruited. Their main baseline characteristics are reported in Table 3. Among them, 48 patients (48.9%) were prescribed TT, 31 (31.6%) received DT and 19 (19.4%) were prescribed DAPT. Mean CHADS2, CHA2DS2-VASc, and HAS-BLED scores were 1.8 ± 1.5, 5.3 ± 1.6, and 2.3 ± 0.5, respectively. After a mean follow-up of 378 ± 15 days, the absolute rates of MACEs, total bleeding, major bleeding, and total events (MACE plus bleeding) were 21.4%, 18.4%, 7.1%, and 39.8%, respectively. In particular, no significant differences across the three therapy groups were identified for both MACEs and total bleedings (Table 4, Fig. 1-3). Likewise, no differences were found in regards to the site of major or minor bleeding across the three therapy categories (Table 5), except for only genitourinary hemorrhages (a kind of minor bleeding) that exhibited a significant difference in distribution among the three groups (0/48 cases in TT patients, 1/31 cases among DT patients and 3/19 cases among DAPT patients; Chi-square test, P = 0.013). Moreover, the lack of significant differences was noticeable in the rate of hemorrhagic relapses by comparing the three therapy groups (Table 5). Likewise, by using the Kaplan-Meier analysis, no significant differences were observed in the survival free from total MACEs and total bleeding events across the three groups (Fig. 4 and 5).

The article "Clinical Relevance of Anticoagulation and Dual Antiplatelet Therapy to the Outcomes of Patients With Atrial Fibrillation and Recent Percutaneous Coronary Intervention With Stent" was retracted in 2025. Reasons: duplicate publication; overlap with earlier publications.

**Table 3:** Baseline Characteristics

	Total (n = 98)	TT (n = 48)	DT (n = 31)	DAPT (n = 19)	P-value
Age(years)	73 ± 7.5	72 ± 7.5	73 ± 8	77 ± 5	0.045
Male gender	44 (45%)	22 (46%)	12 (39%)	10 (53%)	0.62
Hypertension	76 (77.5%)	36 (75%)	27 (87%)	13 (68%)	0.257
Diabetes	34 (35%)	18 (37.5%)	10 (32%)	6 (31.5%)	0.848
Hypercholesterolemia	54 (55%)	27 (56%)	18 (57%)	9 (47%)	0.742
Current smoking	16 (16.5%)	6 (12.5%)	6 (19.3%)	4 (21%)	0.596
Body mass index	27.7 ± 2	27 ± 2	28 ± 2	29 ± 2	0.006
Previous TIA/stroke	13 (13.2%)	10 (20.8%)	2 (6.45%)	1 (5.2%)	0.095
Previous AMI	24 (24.5%)	12 (25%)	6 (19.3%)	6 (31.5%)	0.617
Previous PCI-S/CABG	34 (34.6%)	17 (35%)	10 (32%)	7 (37%)	0.936
Previous major bleeding	4 (4%)	0	2 (6.45%)	2 (10.5%)	0.125
Chronic heart failure	15 (15.3%)	12 (25%)	3 (9.6%)	0	0.022
Chronic kidney disease	28 (28.5%)	13 (27%)	8 (26%)	7 (37%)	0.668
Anemia	12 (11.2%)	1 (2%)	5 (16%)	6 (31.5%)	0.003
LVEF	50 ± 5	50.7 ± 4.7	49.8 ± 6	50 ± 5	0.738
eGFR(MDRD)	68 ± 15.6	72 ± 14	64 ± 14	66 ± 11.5	0.068
AF	90 (92%)	48 (100%)	23 (74%)	19 (100%)	0.0001
Indication for prophylaxis of cardioembolism or venous thromboembolism					
AF	74 (75.5%)	32 (85.4%)	28 (90%)	14 (73.6%)	0,056
Previous VTE/cardiac embolism	3 (3.06%)	3 (6.25%)	0	0	0.199
Dilated cardiomyopathy without AF	1 (1.02%)	0	0	1 (5%)	0.335
Mechanical valve with or without AF	20 (20.4%)	13 (27%)	3 (25.8%)	4 (15.8%)	0.172
Indication for PCI -S requiring antiaggregant agents for a period of 1 month (BMS) or 9 - 12 months (DES)					
Stable exertional angina	30 (30.6%)	12 (25%)	12 (38.7%)	6 (31.6%)	0.432
NSTE-ACS	49 (50%)	23 (48%)	13 (42%)	13 (68.4%)	0.176
Acute STEMI	19 (19.3%)	13 (21%)	6 (19.3%)	0	0.043

Data are reported as absolute number (percentage) or mean ± standard deviation. TT: triple therapy (warfarin + acetylsalicylic acid and clopidogrel); DT: dual therapy (warfarin + acetylsalicylic acid or clopidogrel); DAPT: dual antiplatelet therapy (acetylsalicylic acid + clopidogrel); TIA: transient ischemic attack; AMI: acute myocardial infarction; PCI-S: percutaneous coronary intervention with stent; CABG: coronary artery bypass graft; LVEF: left ventricular ejection fraction; eGFR: estimated glomerular filtration rate; MDRD: Modification of Diet in Renal Disease Study equation; AF: atrial fibrillation; VTE: venous thromboembolism; BMS: bare metal stent; DES: drug-eluting stent; NSTE-ACS: non-ST elevation acute coronary syndrome; STEMI: ST-elevation myocardial infarction.

The article "Clinical Relevance of Anticoagulation and Dual Antiplatelet Therapy to the Outcomes of Patients With Atrial Fibrillation and Recent Percutaneous Coronary Intervention With Stent" was retracted in 2025. Reasons: duplicate publication; overlap with earlier publications.

**Table 4:** Incidence of Adverse Events According to Therapeutic Strategy at Discharge, After a Follow-Up of 1-Year

	Total (n = 98)	TT (n = 48)	DT (n = 31)	DAPT (n = 19)	P-value
Exertional angina	10 (10.2%)	5 (10.4%)	3 (9.6%)	2 (10.5%)	0.993
Total MACE	21 (21.43%)	13 (27.1%)	4 (12.9%)	4 (21%)	0.324
Death from all causes	5 (5.1%)	4 (8.3%)	0	1 (5.3%)	0.258
Total ACS	5 (5.1%)	2 (4.2%)	1 (3.22%)	2 (10.5%)	0.480
Unstable angina	4 (4.08%)	1 (2%)	1 (3.22%)	2 (10.5%)	0.277
Non-fatal AMI	1 (1.02%)	1 (2%)	0	0	0.591
Repeat revascularization	6 (6.12%)	2 (4.2%)	3 (9.6%)	1 (5.3%)	0.599
Stent thrombosis	1 (1.02%)	1 (2%)	0	0	0.591
DVT/PE	3 (3.06)	3 (6.25%)	0	0	0.199
Stroke/TIA	1 (1.02%)	1 (2%)	0	0	0.591
Total bleeding	18 (18.4%)	8 (16.66%)	6 (19.35%)	4 (21%)	0.903
Major	7 (7.1%)	4 (8.3%)	2 (6.45%)	1 (5.3%)	0.893
Minor	11 (11.33%)	4 (8.3%)	4 (12.9%)	3 (15.8%)	0.642

Data are reported as absolute number (percentage). TT: triple therapy (warfarin + acetylsalicylic acid and clopidogrel); DT: dual therapy (warfarin + acetylsalicylic acid or clopidogrel); DAPT: dual antiplatelet therapy (acetylsalicylic acid + clopidogrel); MACE: major adverse cardiovascular event; ACS: acute coronary syndromes; AMI: acute myocardial infarction; TIA: transient ischemic attack; DVT: deep vein thrombosis; PE: pulmonary embolism.

**Figure 1:** Distribution of total MACEs across the three treatment groups. No significant differences were found between groups as regards the frequency of total MACEs (21%, 12.9% and 27.1% in DAPT, DT and TT groups, respectively; Chi-square test, P = 0.324). TT: triple therapy (warfarin + acetylsalicylic acid (ASA) and clopidogrel); DT: dual therapy (warfarin + ASA or clopidogrel); DAPT: dual antiplatelet therapy (ASA + clopidogrel); MACE: major adverse cardiovascular event; pts, patients.

**Figure 2:** Distribution of total bleeding events across the three treatment groups. No significant differences were found between groups as regards the frequency of total bleeding events (21%, 19.35% and 16.6% in DAPT, DT and TT groups, respectively; Chi-square test, P = 0.903). TT: triple therapy (warfarin + acetylsalicylic acid (ASA) and clopidogrel); DT: dual therapy (warfarin + ASA or clopidogrel); DAPT: dual antiplatelet therapy (ASA + clopidogrel); pts: patients.

The article "Clinical Relevance of Anticoagulation and Dual Antiplatelet Therapy to the Outcomes of Patients With Atrial Fibrillation and Recent Percutaneous Coronary Intervention With Stent" was retracted in 2025. Reasons: duplicate publication; overlap with earlier publications.

**Figure 3:** The type of antithrombotic regimen at the time of major bleeding is highlighted. Four out of seven major bleeding events occurred in the course of TT regimen; however, no significant difference (Chi square test, P = 0.893) was demonstrated for the incidence of major bleeding across the three treatment groups, among whom the TT group was the most numerous (48 pts vs. 31 pts in the DT group and only 19 patients in the DAPT group). TT: triple therapy (warfarin + acetylsalicylic acid (ASA) and clopidogrel); DT: dual therapy (warfarin + ASA or clopidogrel); DAPT: dual antiplatelet therapy (ASA + clopidogrel); pts: patients.

**Table 5:** Sites of Bleeding Found During 1-Year Follow-Up

	Total no. of pts (n = 98)	TT (n = 48)	DT (n = 31)	DAPT (n = 19)	P-value
Bleeding events (major and minor)	18 (18.4%)	8 (16.66%)	6 (19.35%)	4 (21%)	0.903
Major bleeding events					
Total	7 (7.1%)	4 (8.3%)	2 (6.45%)	1 (5.2%)	0.893
Intracranial	2 (2.04%)	1 (2.1%)	1 (3.2%)	0	0.735
Gastrointestinal	2 (2.04%)	1 (2.1%)	1 (3.2%)	0	0.735
Genitourinary	2 (2.04%)	1 (2.1%)	0	1 (5.2%)	0.442
Other (iliopsoas hematoma)	1 (1.02%)	1 (2.1%)	0	0	0.591
Minor bleeding events					
Total	11 (11.33%)	4 (8.3%)	4 (12.9%)	3 (15.8%)	0.642
Nose	7 (7.1%)	4 (8.3%)	3 (9.6%)	0	0.394
Genitourinary	4 (4.1%)	0	1 (3.2%)	3 (15.8%)	0.013
Relapses of minor bleeding					
Minor bleeding events > 1 in the same patient	8 (8.16%)	5 (10.4)	2 (6.45%)	1 (5.26%)	0.719

Data are reported as number (percentage). pts: patients; TT: triple therapy (warfarin + acid acetylsalicylic acid and clopidogrel); DT: dual therapy (warfarin + acid acetylsalicylic or clopidogrel); DAPT: dual antiplatelet therapy (acetylsalicylic acid + clopidogrel).

**Figure 4:** The Kaplan-Meier curve is used to compare the respective probabilities of being involved by an MACE across the three antithrombotic treatment groups. No significant differences across the three pharmacologic regimens were observed in the survival free from total MACE over a 1-year follow-up (log-rank test, P = 0.284). DAPT: dual antiplatelet therapy (acetylsalicylic acid (ASA) + clopidogrel); DT: dual therapy (warfarin + ASA or clopidogrel); TT: triple therapy (warfarin + ASA and clopidogrel).

**Figure 5:** The Kaplan-Meier curve is used to compare the respective probabilities of being involved by one or more bleeding events (major or minor) across the three antithrombotic treatment groups. No significant differences across the three pharmacologic regimens were observed in the survival free from total bleeding events over a 1-year follow-up (log-rank test, P = 0.955). DAPT: dual antiplatelet therapy (acetylsalicylic acid (ASA) + clopidogrel); DT: dual therapy (warfarin + ASA or clopidogrel); TT: triple therapy (warfarin + ASA and clopidogrel).

The article "Clinical Relevance of Anticoagulation and Dual Antiplatelet Therapy to the Outcomes of Patients With Atrial Fibrillation and Recent Percutaneous Coronary Intervention With Stent" was retracted in 2025. Reasons: duplicate publication; overlap with earlier publications.

In our experience, the TT duration never exceeded the limit of 3 months. Therefore, in our case records, there were a number of patients for whom DT was planned as a therapeutic starting strategy (for AF or other conditions entailing thromboembolic risk among patients also requiring simultaneous prophylaxis of intra-stent thrombosis) together with another group of patients, where DT with warfarin plus an antiplatelet drug (ASA or clopidogrel) represented the continuation of the original TT scheme. The therapy was either stopped after 1 month if a BMS had been implanted or was interrupted after a variable period (extending from 1 to 3 months) if a DES had been used. In this scenario, AF cases that occurred after stent implantation (i.e., 20 patients) were significantly less frequent compared to those in which AF occurrence had preceded the percutaneous coronary procedure (i.e., 78 patients) (Chi-square test, P < 0.0001). However, although the risk of bleeding might appear more pronounced in the cases of AF that had arisen after PCI-S because of the higher expected number of DES implants in this subset and because of the related need for prolonged DAPT, the incidence of bleeding events in the two subsets was comparable (P = 0.9116) (Table 6).

**Table 6:** Frequency of the Bleeding Events Within the Two AF Subsets Enrolled in the Study: AF Pre-Existing With Respect to PCI-S (78 Patients) or Arisen After PCI-S (20 Patients)

	AF already present before the interventional procedure of coronary stenting (no. 78 patients)	AF arisen during the year following the interventional procedure of coronary stenting (no. 20 patients)	P-value (Chi-square test)
Bleeding events	14	4	0.9106

AF: atrial fibrillation; PCI-S: percutaneous coronary intervention with stent implantation.

Moreover, importantly, all the four major bleeding events reported among patients assigned to TT occurred while administering the triple drug combination. Actually, in regards to the two major bleeding events signaled in the DT group, they involved patients who had been assigned from the first moment to DT, due to their HAS-BLED score that indicated they were at high risk of bleeding. Indeed, bleeding did not occur in cases when DT was administered as a continuation of the original TT after the latter had been stopped. In fact, no case of major bleeding was found in the timeframe subsequent to the switch from TT to DT.

## Discussion

The present analysis focused on outpatients, each of whom had experienced a condition requiring OAC with warfarin (AF, deep venous thrombosis, history of ascertained or suspected cardioembolism, or mechanical cardiac prosthesis). This need for OAC was complicated by the concomitant need for antiaggregant agents, since every patient had recently undergone a percutaneous transluminal coronary angioplasty (PTCA) with stent implantation, thus requiring a dual antiplatelet regimen, according to the current guidelines [2, 3]. Therefore, two different scenarios were represented in our study, depending on whether the condition requiring OAC had preceded the stenting procedure or had taken place after the PCI-S. In the first case (i.e., AF preceding the PCI), the adoption of BMS was consistently preferred on occasion of the subsequent angioplasty with stenting, considering that this type of coronary prosthesis does not cause a sustained loss of endothelium, thus requiring a relatively short duration (usually, 1 month) of the DAPT (ASA + thienopyridine) for the prophylaxis of intra-stent thrombosis. This is very important because with this method, the combined regimen of an anticoagulant joined with a dual antiplatelet treatment is unlikely to generate a high amount of bleeding events, given the relatively short duration (not more than 1 month) of the DAPT as scheduled by this protocol. Instead, in the second case, the AF occurs after the patient has already undergone a PCI-S that (in high income countries) generally entails the use of a DES, i.e., a stent that elutes an immunosuppressant drug. In this setting, very challenging problems arise because in the case of DES, the prophylaxis of the intra-stent thrombosis with DAPT should be conducted for at least 12 months [12, 13], which amplifies the risk that a possible combination regimen comprising the OAC can result in bleeding complications. This concern is the reason for the current trend to maintain TT for a relatively short period (1 - 3 months in our experience) and then convert it into a less demanding regimen, namely, a hybrid protocol that provides for a single antiplatelet agent (e.g., ASA or clopidogrel) in addition to warfarin or, alternatively, the maintenance of only DAPT. As presented in the “Results”, the three antithrombotic regimens of TT, DT, and DAPT that we used in our study exhibited comparable efficacy and safety throughout the prescribed period of follow-up (mean duration among the 98 patients retrospectively examined: 378 ± 15.7 days). The absolute 1-year rates of major bleeding with TT, DT, and DAPT were 8.3%, 6.45%, and 5.2%, respectively (Chi-square test, P = 0.893). By comparing the three different therapeutic regimens tested in our study (TT, DT and DAPT), no significant difference was detected regarding the incidence of MACEs (ACSs, need for percutaneous or surgical revascularization, or ischemic stroke) or all-cause mortality. In regards to this aspect, the literature data are somewhat contradictory. In fact, based on the results of the ACTIVE-W study [1], there is documentation of higher efficacy of oral warfarin compared to combination therapy clopidogrel + ASA for the prevention of the ischemic stroke in AF patients. In the above mentioned study, the clopidogrel plus ASA group showed significantly more MACEs, such as stroke, non-central nervous system systemic embolism, myocardial infarction, or vascular death compared to those who received oral warfarin (P = 0.0003). Thus, the study was stopped early owing to the clear superiority of the warfarin therapy. By contrast, there are several studies in the literature that demonstrate a substantially comparable preventive efficacy against MACEs exerted by the three abovementioned regimens [8, 14]. Moreover, recent data from the prospective, randomized WOEST study [15] have even shown superior efficacy of DT (with warfarin plus clopidogrel) over TT in regards to the occurrence of MACEs. In addition, in their recent study concerning the prospective, multicenter WARfarin and coronary STENTing (WAR-STENT) registry, conducted among patients with chronic AF and recent coronary angioplasty with stenting (mostly using BMSs), Rubboli et al [16] detected no evidence of superiority of the TT regimen compared to the simplified scheme consisting of a single antiplatelet agent (ASA or clopidogrel) added to an OAC (warfarin). Indeed, in this study, no differences in terms of antithrombotic efficacy were evident, based on the comparison between TT, DT (i.e., warfarin supplemented by either ASA or clopidogrel) and DAPT with ASA and clopidogrel. Furthermore, in the above mentioned study, even an alleged and greatly feared high incidence of major bleeding was not proven in the group of patients assigned to TT scheme. At 12 months, in fact, the frequency of major bleeding events was 4% (14/339 patients), 5% (1/20 patients) and 2% (1/42 patients) in the TT, DT and DAPT groups, respectively.

The article "Clinical Relevance of Anticoagulation and Dual Antiplatelet Therapy to the Outcomes of Patients With Atrial Fibrillation and Recent Percutaneous Coronary Intervention With Stent" was retracted in 2025. Reasons: duplicate publication; overlap with earlier publications.

In patients requiring both the OAC and the prophylaxis of intra-stent thrombosis, our study did not show a superiority of TT regimen compared to alternative schemes consisting of DAPT or combined administration of warfarin with only one antiplatelet agent with regard to efficacy outcomes (MACEs and mortality from all causes) as well as for the safety endpoints (bleeding events). Therefore, our study adds to the already quite numerous series [8, 14-16] of preexisting investigations that have disavowed the alleged higher anti-ischemic protection through the practice of adding two, rather than one, antiplatelet agent on top of OAC in patients with AF and recent PCI-S. Really, not even the recent official guidelines provide convincing evidence that TT has better therapeutic efficacy in this clinical setting, considering that European and American position documents categorize recommendations for TT as “Level of Evidence C” [17, 18].

### Study limitations

The small sample size and its retrospective observational design are the main limitations of the study. Thus, possible indication biases are likely to have occurred, for example, due to the allocation to the TT group of patients presenting the most severe clinical picture and the highest CHA_2_DS_2_-VASc score. In this way, due to the lack of balance of clinical characteristics across the three groups, the possible higher antithrombotic efficacy of TT may have been hidden or undersized. Moreover, in the present study, the significance of the anti-ischemic protective effect and the potential risk for bleeding of other drug combinations (prasugrel + ASA, ticagrelor + ASA) were not explored, because the data harvested from our outpatient population date back a few years ago when these novel antiplatelet agents were not used in a routine manner at our institute, whilst the new OACs, alternative to warfarin (dabigatran, rivaroxaban, apixaban, etc.) [19] had not been validated yet for clinical use.

### Conclusions

Based on our retrospective study, the three antithrombotic regimens TT, DT, and DAPT showed comparable efficacy and safety. Further studies with larger sample sizes, preferably modeled as randomized clinical trials, should be planned for comparing the various feasible regimens (with anticoagulant plus single or DAPT or consisting of the association of two platelet antiaggregants) among patients with indication for OAC and the concomitant need for protection against stent thrombosis due to recent PCI-S.
